# Calycosin Ameliorates Bleomycin-Induced Pulmonary Fibrosis via Suppressing Oxidative Stress, Apoptosis, and Enhancing Autophagy

**DOI:** 10.1155/2022/9969729

**Published:** 2022-10-11

**Authors:** Haoge Liu, Xiaoxu Bai, Wan Wei, Zhipeng Li, Zhengju Zhang, Weili Tan, Bin Wei, Hantao Zhao, Yang Jiao

**Affiliations:** ^1^Graduate School, Beijing University of Chinese Medicine, Beijing, China; ^2^Department of Respiratory, Fangshan Hospital Affiliated to Beijing University of Chinese Medicine, Beijing, China; ^3^Department of Geratology, Dongfang Hospital Affiliated to Beijing University of Chinese Medicine, Beijing, China; ^4^Department of Respiratory, Dongfang Hospital Affiliated to Beijing University of Chinese Medicine, Beijing, China

## Abstract

Calycosin (CA) is a flavonoid extracted from the root of *Astragalus membranaceus* and has antioxidant, anti-inflammation, and antiapoptosis properties. The objective of this study was to investigate the efficacy of CA in protecting against pulmonary fibrosis. CA (14 mg/kg) and SB216763 (20 mg/kg) were administrated to bleomycin-induced pulmonary fibrosis mice for 3 weeks. The results concluded that CA alleviated the inflammation and collagen deposition in pulmonary fibrosis. In addition, CA reduced MDA level, enhanced SOD and TAC activities, and increased the activity of the Nrf2/HO-1 pathway. CA also regulated the expressions of apoptosis-related proteins. Moreover, CA enhanced autophagy via upregulating LC3, beclin1, PINK1, and reducing p62. CA also increased expression of LAMP1 and TFEB, and inhibited the release of lysosome enzymes from ruptured lysosomes. These results provide new evidence that CA protects against pulmonary fibrosis through inhibiting oxidative stress and apoptosis. In addition, autophagy abnormality and lysosome dysfunction are restored by CA.

## 1. Introduction

Idiopathic pulmonary fibrosis (IPF) is a devastating lung disease of unknown aetiology characterized by progressive fibrosing interstitial pneumonitis, fibroblast proliferation, and excessive extracellular matrix production [1]. The median survival duration of IPF averages to 3–5 years after diagnosis. IPF occurs primarily in the elderly men, and most patients have a history of smoking. Although nintedanib and pirfenidone are currently approved by the Food and Drug Administration as pharmacological therapies for IPF, neither of them can improve survival rates among patients with IPF [2, 3]. Lung transplantation is the only cure for IPF patients. There is an urgent need to find new therapeutic drugs for IPF treatment. The lung is a delicate and essential organ directly exposed to air and its constituent pathogens, airborne irritants, and hazardous pollutants. Oxidative stress contributes to pulmonary fibrosis by multiple mechanisms. Hyperoxia-induced oxidative damage results in alveolar epithelial cell apoptosis [4]. Mitochondrial reactive oxygen species (mtROS) generation by mitochondrial complex III has been shown to enhance the process of differentiation into the myofibroblast phenotype [5]. Studies identified that intermittent hypoxia-mediated oxidative stress accentuated bleomycin (BLM)-induced pulmonary fibrosis [6]. The genetic knockout of Nrf2 exacerbates experimental pulmonary fibrosis of mice. In addition, the activation of Nrf2/HO-1 pathway suppresses epithelial-mesenchymal transition in pulmonary epithelial cells [7]. Thus, targeting the oxidative stress may serve as a therapeutic strategy for pulmonary fibrosis.

Autophagy is a process that relies on lysosomes to degrade damaged organelles or proteins. Mitochondrial autophagy is a selective form of autophagy. The inactivation of autophagy results in the accumulation of proteins and morphologically abnormal mitochondria [8]. In addition, ROS leads to mitochondrial damage, which in turn leads to more ROS release. Therefore, aberrant autophagy is suggested as a pathological driver of pulmonary fibrosis [9]. A previous study indicated that impaired autophagy was observed in the lungs of BLM-treated mice [10]. Moreover, Atg4b gene deletion exacerbated collagen accumulation and promoted excessive extracellular matrix-related gene expression [11]. Targeting autophagy may be an effective approach for inhibiting pulmonary fibrosis. Kim et al. reported that interleukin-37 inhibited oxidative stress-induced alveolar epithelial cell (AEC) death via transforming growth factor-*β*1 signaling through enhancement of autophagy [12]. Kurita et al. suggested that pirfenidone inhibited the myofibroblast differentiation through autophagy/mitophagy activation and reducing mitochondrial ROS via PDGFR-PI3K-Akt pathway [5].

The aetiology and molecular mechanisms of pulmonary fibrosis is not well elucidated. Considerable attention has been invested in the search for novel efficient natural drugs of plant origin for pulmonary fibrosis. Calycosin, one of the flavonoids, is extracted from the root of *Astragalus membranaceus*. It was previously demonstrated that CA could attenuate pulmonary fibrosis [13]. One study indicated that after the oral administration of pulmonary rehabilitation mixture (124.4 *μ*g/g of CA), the AUC_0-*t*_, AUC_0-∞_, and *t*_1/2_ of CA in pulmonary fibrosis rats increased markedly compared to normal rats [14]. Calycosin has the potential to be developed into an antifibrotic drug. However, the specific therapeutic mechanism of CA requires further investigations. In this study, BLM was used to establish rodent models to mimic the pathologic features of pulmonary fibrosis. We aimed to evaluate whether CA could mitigate BLM-induced pulmonary fibrosis by reducing oxidative stress and regulating apoptosis and autophagy.

## 2. Materials and Methods

### 2.1. Chemicals and Regent

Calycosin was obtained from Chengdu Must Bio-Technology Co., Ltd. (Chengdu, China; cat: A0514); its purity was ≥99%. Bleomycin was supplied by Fresenius Kabi (Lake Zurich, USA). SB216763 (SB) was purchased from MedChem Express (Shanghai, China; cat: HY-12012).

### 2.2. Animals

All mice experiments were approved by and performed in accordance with the guidelines of the Animal Experimental Ethical Committee of Beijing University of Chinese Medicine. This study included 40 C57BL male mice weighing 22 ± 2 g each. The seven-week-old mice were purchased from Beijing Vital River Laboratory Animal Technology Co., Ltd. (Beijing, China). The mice were housed under laboratory conditions. The temperature was kept at 22–26°C, and the ambient humidity was kept at 50%–60%. Food and water were freely available to the mice.

### 2.3. Animal Treatment

Forty mice were randomly divided into 4 groups: normal control (NC) group, BLM group, CA group, and SB group. After one week of adaptive feeding, the mice were all anesthetized with isoflurane inhalation (5% isoflurane induction) to modelling. Except for the NC group, all mice were instilled BLM (2 U/kg) solution from the airway as described previously [15]. The NC group was administered the same amount of physiological saline. One day later, the mice in each group were treated as follows.

NC and BLM groups: mice were administered with physiological saline by gavage once a day for 21 days and the vehicle (25% dimethyl sulfoxide, 25% polyethylene glycol, and 50% saline) was administered by intraperitoneal injection twice a week.

CA group: mice were administered with CA (14 mg/kg) [13] by gavage once a day for 21 days and the vehicle (25% dimethyl sulfoxide, 25% polyethylene glycol, and 50% saline) was administered by intraperitoneal injection twice a week.

SB group: mice were administered with physiological saline by gavage once a day for 21 days and SB216763 (20 mg/kg) dissolved in the vehicle was administered by intraperitoneal injection twice a week [16]. SB216763, one of the glycogen synthase kinase 3*β* inhibitor, can promote autophagy and inhibit apoptosis [17].

The body weight of each mouse was measured every 3 days. All mice were euthanized using isoflurane at the end of 21 days.

### 2.4. Histological Staining

For hematoxylin-eosin (HE) staining, the left lung samples were fixed immediately with 4% paraformaldehyde, paraffin-embedded, and sectioned at 4 *μ*m. The sections were then counterstained with hematoxylin (15 min) and eosin (5 min). The tissue sections were stained with Masson using the corresponding kit (Solarbio Life Sciences, Beijing, China). Semiquantitative analysis of inflammation was performed using Alveolitis and Ashcroft scores, respectively. The area of positive staining for Masson trichrome was measured, and then compared to the total area as a ratio using ImageJ software (ImageJ Software Inc., Marlyand, USA).

### 2.5. Immunohistochemistry Analysis

Immunohistochemistry was performed as previously described [18]. In short, after dewaxing and rehydration, the slides were immersed in microwave-pretreated boiling citrate buffer (0.01 M, pH 8.0) for antigen repair. After cooling at room temperature (21°C), 3% H_2_O_2_ was added to deactivate endogenous peroxidase. The slides were washed in phosphate buffer solution and incubated with blocking serum (10% nonimmune goat serum) to block nonspecific immunolabeling at room temperature (21°C). Primary antibodies were incubated with the slides overnight at 4°C. Slides were then incubated with the appropriate secondary antibodies. After rinsing with phosphate buffer solution, the sections were visualized with diaminobenzidine and counterstained with hematoxylin. Neutral gum was used for sealing, and all the sections were photographed under an Olympus BX50F4 light microscope (Olympus, Center Valley, PA).

### 2.6. Superoxide Dismutase (SOD), Total Antioxidant Capacity (TAC), and Malondialdehyde (MDA) Measurements

Serum was separated by low‐speed centrifugation (3000 r/min) for 15 minutes. The levels of MDA, SOD, and TAC in serum were detected with an automatic analyzer (Biochemical analyzer BS-200, Mindray, China). The operation process was carried out according to the manufacturer's instructions.

### 2.7. Western Blot Assay

Briefly, lung tissues were homogenized and the proteins were extracted in tissue lysis buffer. Total proteins were quantified with bicinchoninic acid protein assay kits (MD913053; MDL, Beijing, China) following the manufacturer's instructions. 20 *μ*g proteins per sample were separated by sodium dodecyl sulfate-polyacrylamide gel electrophoresis on 10% gels and transferred to polyvinylidene difluoride membranes. The membrane was blocked for 2 hours by 5% skimmed milk in Tris-buffered saline at room temperature (21°C). For antibody staining, samples were incubated with primary antibodies at 4°C overnight including anti-LC3A/B (Affinity, AF5402, 1 : 1000), anti-SQSTM1/p62 (Affinity, AF5384, 1 : 1000), anti-Beclin 1 (Affinity, AF5384, 1 : 1000), anti-LAMP1 (Affinity, AF5182, 1 : 1000), anti-HO-1 (Affinity, DF7033, 1 : 1000), anti-PINK1 (Affinity, AF5393, 1 : 1000), goat anti-rabbitIgG-HRP (Affinity, S0001, 1 : 1000), goat anti-rabbitIgG-FITC (Affinity, S0008, 1 : 1000), rabbit anti-collagenalpha-1 (Bioss, bs-20124R, 1 : 1000), and rabbit anti-Legumain (Bioss, bs-3907R, 1 : 1000). Membranes were incubated with appropriate secondary antibody (MDL, MD932477, 1 : 10,000) for 1 hour at room temperature (21°C). The protein bands were visualized by using the enhanced chemiluminescence detection system (ThermoFisher, Waltham, MA) and were quantified using a ChemiDoc Imaging System (Bio-Rad, USA). All of the determinations were performed independently and repeated three times.

### 2.8. Transmission Electron Microscopy

Transmission electron microscopy (TEM) was performed to observe the autophagy-related structure. Lung tissues were post-fixed in 1% osmium tetroxide for 3 hours. After dehydration with graded ethanol and acetone, samples were embedded in Spurr, sliced into 70 nm thick pieces, stained with uranyl acetate and lead citrate, and observed using TEM (JEM-1400, JEOL, Tokyo, Japan). The number of autolysosomes was evaluated at 20,000×.

### 2.9. RNA Isolation and Quantitative Real-Time Polymerase Chain Reaction (PCR) Analysis

Total RNA was extracted using Trizol (cat. No. 10296028, TRIzol, Invitrogen) following manufacturer's instructions. The RNA concentration and purity were determined using an Eppendorf Biophotometer (Eppendorf Company, Hamburg, Germany). The total RNA was then converted into cDNA using Superscript III RT-PCR kit (Invitrogen, cat no. 11752050). The primers used were as follows: Nrf2: forward 5′-ACTCAAATCCCACCTTAAACAC-3′, reverse 5′-GTCACAGCCTTCAATAGTCCC-3′; XIAP: forward 5′-ATATGAAGCACGGATCGTTA-3′, reverse 5′-CTCCTCCACAGTGAAAGCA-3′; Bax: forward 5′-AGGGTTTCATCCAGGATCGAGCA-3′, reverse 5′-CAGCTTCTTGGTGGACGCATC-3′; Bcl-2: forward 5′-ACTTCTCTCGTCGCTACCGTC-3′, reverse 5′-CCCCATCCCTGAAGAGTTCCT-3′; TFEB: forward 5′-AGTGGTCTTGGGCAAATCCCTTCT-3′, reverse 5′-TGGTTCGGGCTCCCTGTAGTCG-3′;*β*-actin: forward 5′-CCAGCCTTCCTTCTTGGGTA-3′, reverse 5′-CAATGCCTGGGTACATGGTG-3′.*β*-actin was chosen as a control, and gene expression levels were quantified by the 2^−ΔΔCT^ method.

### 2.10. Statistical Analysis

Statistical analysis was performed using GraphPad Prism 8.0 software (GraphPad Software, San Diego, USA). The data were presented as mean ± SD. One-way ANOVA followed by Tukey's post hoc test were used for intragroup and intergroup comparisons. Any difference was considered significant when *P* < 0.05.

## 3. Results

### 3.1. The Effect of CA on BLM-Induced Pulmonary Fibrosis

To explore the effect of CA on pulmonary fibrosis, lung tissues were analyzed by HE and Masson staining. In Figure 1(a), HE showed severe damage of lung structure after BLM administration. The walls of the alveoli and the alveolar septum were thickened and a large degree of inflammatory cell infiltration was observed. Calycosin and SB treatment attenuated these changes, while the lung injury score (*P* < 0.01) and Ashcroft score (*P* < 0.01) were significantly decreased (Figures 1(d) and 1(e)). Masson staining showed that interstitial fibrosis and disruption of lung structure occurred in BLM-induced mice. However, treatment with CA and SB markedly reduced collagen deposition (Figures 1(b) and 1(f), *P* < 0.01). Collagen I is one of the major collagen proteins of the extracellular matrix, which is an important biomarker of pulmonary fibrosis. The expression of collagen I was tested by immunohistochemistry. Compared with that in the NC group, the expression of collagen I was significantly higher in the BLM group. By contrast, the expression of collagen I was reduced in the lung tissues of the CA group and SB group (Figure 1(c)). Taken together, our data indicates that CA was effective against the progression of pulmonary fibrosis.

### 3.2. The Effect of CA on Oxidant/Antioxidant Markers in BLM-Induced Pulmonary Fibrosis

Oxidative stress is an important contributor to the pathogenesis of pulmonary fibrosis. The activities of antioxidant factors, SOD (*P* < 0.01) and TAC (*P* < 0.01), in the serum of BLM-induced mice were significantly lower than that of the NC group, while CA administration was observed to increase both SOD (*P* < 0.01) and TAC (*P* < 0.01) levels (Figures 2(b) and 2(c)). In addition, the level of serum MDA, an index of lipid peroxidation was significantly decreased in the CA group compared with the BLM group (Figure 2(a), *P* < 0.05). The Nrf2 and HO-1 are excellent indicators of oxidation and antioxidation processes. This study shows that the relative expression of Nrf2 mRNA expression was decreased with BLM treatment (*P* < 0.01), while CA (*P* < 0.01) and SB (*P* < 0.01) could help increase Nrf2 mRNA expression in the lung (Figure 2(d)). HO-1 was detected by western blotting. BLM administration appears to decrease HO-1 expression, but it was not significant compared to the NC group. In addition, the HO-1 expression in BLM-induced mice was significantly increased with CA (*P* < 0.05) and SB (*P* < 0.01), when compared to the BLM group. In summary, these data demonstrate that CA alleviated the oxidative stress induced by BLM.

### 3.3. The Effect of CA on Apoptosis in BLM-Induced Pulmonary Fibrosis

Oxidative stress generally induces apoptosis. Therefore, the expression of apoptosis-related markers was also measured. Bcl-2 is an antiapoptotic protein while Bax enhances apoptosis. We found that the expression of Bcl-2 in the BLM group was decreased as compared to the NC group (*P* < 0.01), while CA treatment could restore Bcl-2 expression (*P* < 0.01). Moreover, Bax expression was much activated in the BLM group (*P* < 0.01), while CA treatment (*P* < 0.01) noticeably decreased Bax content (Figures 2(a) and 2(b)). The overexpression of XIAP could decrease apoptosis. While BLM was shown to inhibit XIAP expression (*P* < 0.01), a nonsignificant recovery of XIAP expression was observed in the CA group. HK-2 is also an antiapoptotic protein. HK-2 downregulation by BLM was confirmed in the lung tissue by immunohistochemical staining, while CA was observed to significantly increase HK-2 expression. These data suggest that CA protects against pulmonary fibrosis by inhibiting apoptosis (see Figure 3).

### 3.4. The Effect of CA on Autophagy in BLM-Induced Pulmonary Fibrosis

To explore whether CA improved pulmonary fibrosis via autophagy, we measured the expression of autophagy-related proteins in fibrotic lung tissues. As shown in Figures 4(a)‒4(c), the level of beclin 1 in the BLM group was much lower than that of the NC group (*P* < 0.01), but was increased with SB treatment (*P* < 0.01). The level of PINK1 in the BLM group was higher than that of the NC group (*P* < 0.01), and interestingly, the expression level of PINK1 was further elevated by CA (*P* < 0.01). Unexpectedly, no significant differences in LC3-II and LC3-II/LC3-I were observed between the NC and BLM groups. Nevertheless, CA significantly increased (*P* < 0.01) the conversion of LC3-I to LC3-II (Figures 4(d) and 4(e)). p62 accumulation levels are proportional to the autophagic impairment. Compared with the NC group, the expression level of p62 in the BLM group was significantly increased (*P* < 0.01). After treatment with CA (*P* < 0.01) and SB (*P* < 0.01), p62 expression was obviously decreased (Figure 4(f)). p62 immunohistochemical staining was found consistent with western blot analysis (Figure 4(g)). The morphological changes of the lung tissue were observed using TEM. Compared with the NC group, the cells from the BLM group exhibited few autophagic vesicles, while numerous mitochondria were swollen and enlarged (Figure 5). After administration of CA and SB, the numbers of intracellular autophagosome and autolysosome were increased. Taken together, this data indicated that CA promotes autophagy, which may be responsible for its effects in the alleviation of pulmonary fibrosis.

### 3.5. Effect of CA on Lysosome Injury in BLM-Induced Pulmonary Fibrosis

Lysosomes are the degradation centres of the autophagy pathway. In our study, we used LAMP1, legumain, and TFEB to monitor lysosomal function. Compared with the NC group, the expression level of LAMP1 was inhibited in the BLM group (*P* < 0.05), but significantly upregulated in both CA (*P* < 0.01) and SB (*P* < 0.01) groups. As shown in Figure 6(c), the expression level of legumain in the BLM group was increased (*P* < 0.01), while treatment with CA decreased legumain protein expression (*P* < 0.05). However, SB administration failed to decrease the expression of legumain. The findings were confirmed by immunohistochemistry of legumain (Figure 6(e)). TFEB is the master regulator of lysosome biogenesis. TFEB mRNA was decreased after BLM administration (*P* < 0.01). However, CA (*P* < 0.01) and SB (*P* < 0.01) reversed the BLM-induced reduction of TFEB (Figure 6(d)). Overall, CA alleviates BLM-induced lysosomal damage.

## 4. Discussion

Calycosin, the most abundantly found isoflavone in *Astragalus*, is a promising antifibrotic agent. It showed promising antioxidant [19], anti-inflammatory [20], and antiapoptotic abilities [21]. Many studies have demonstrated that CA presents as a promising drug for the treatment of organ fibrosis. CA has the potential to be developed into an antifibrotic drug. Zhang et al. suggested that CA mitigated liver fibrosis induced by intraperitoneal injection of CCl4 by reducing oxidative stress via JAK-STAT3 pathway [22]. Elsherbiny et al. indicated that CA ameliorated renal glomerulosclerosis and interstitial fibrosis in diabetes via modulating oxidative stress by IL33/ST2 signaling [23]. Wang et al. reported that CA significantly inhibited the expression and deposition of collagen I and collagen III in cardiac fibrosis [24]. The cardioprotective effects of CA were mediated through upregulations of the PI3K/AKT pathway. In pulmonary fibrosis, Liu et al. reported that CA treatment ameliorated the severity of the lung tissue damage of the fibrosis mice model induced by BLM [13]. Moreover, CA reduced transforming growth factor-*β*1-inducedepithelial-mesenchymal transition in AECs. The therapeutic effects of CA were associated with the AKT/GSK3*β* pathway. However, further studies are required to elucidate the biological mechanisms underlying the protective effect of CA. In this study, we attempted to explore the protective effects of CA on BLM-induced pulmonary fibrosis via suppressing oxidative stress, apoptosis, and enhancing autophagy.

Pulmonary fibrosis is a progressive fibroproliferative disorder associated with high mortality and poor prognosis. In recent years, natural products have attracted great attention for medicinal purposes, including pulmonary fibrosis. Prior studies have demonstrated that quantities of natural products exert preventive and therapeutic effects on pulmonary fibrosis through various mechanisms. There is increasing evidence that oxidative stress contributes to pathogenesis of pulmonary fibrosis. Our previous study showed that ROS could result in significant damage to alveolar epithelium, favoring the progression of pulmonary fibrosis [25]. The oxidative stress can be estimated by the levels of ROS, MDA, SOD as well as the activity of GSH-Px. Plants are significant sources of natural antioxidants, and the antioxidant activity of phenolic compounds has been widely recognized. Hesperetin [26], adelmidrol [27], and curcumin [28] upregulated the expression of GSH, SOD, and CAT, reduce MDA and ROS production, and suppress bleomycin- and silica-induced oxidative damage in pulmonary fibrosis. Nrf2 is the master activator for most of the antioxidant enzymes, and its expression was lower in the fibroblasts and myofibroblasts of patients with IPF [29]. Bergenin improve pulmonary fibrosis by inducing the activation of Nrf2 to relieve oxidative stress and reduce the deposition of the extracellular matrix [30]. Some studies indicated that CA showed good capability against oxidative stress [31], which protected cells from injury. However, there has been no report about the antioxidant activity of CA in pulmonary fibrosis thus far. In the present study, increasing MDA expression and impaired antioxidant enzyme activities of SOD and TAC were observed in pulmonary fibrosis mice. CA reduced MDA levels and increased SOD and TAC activities. HO-1 is a critical downstream antioxidant enzyme of Nrf2. Our results showed that there was a significant increase in the Nrf2 mRNA levels and HO-1 protein levels after CA administration.

As known, AEC injury is an essential first step in the pathogenesis of pulmonary fibrosis. Excessive ROS production can damage cellular components, thus triggering the apoptosis of AECs [32]. Apoptosis mainly involves two major pathways: the mitochondrial apoptotic pathway and the death receptor pathway. In the mitochondrial apoptosis pathway, apoptosis is the result of downregulation of mitochondrial membrane potential, and cytochrome C is released from mitochondria into the cytosol [33]. Bcl-2 family proteins are key regulators of apoptosis. Bax, one of the Bcl-2 family members, promotes apoptosis by damaging mitochondrial membrane integrity, whereas Bcl-2 inhibits apoptosis by maintaining the integrity of the mitochondrial membrane [34]. The X-linked inhibitor of apoptosis protein has also been implicated in mitochondrial apoptosis [35]. It inhibits apoptosis mainly by interacting directly with caspases to inhibit them. HK-2 is a structural protein of mPTP, which is essential for maintaining the integrity of mitochondrial membrane structure and mitochondrial membrane potential [36]. After baicalin administration, the TUNEL-positive cells of BLM-treated rats were significantly decreased. Moreover, baicalin increased Bcl-2, and suppressed Bax protein expression in rat lung tissues [37]. Glycyrrhizic acid treatment remarkably ameliorated BLM-induced pulmonary fibrosis by inhibiting proliferation of fibroblast cells and promoted apoptosis in vitro [38]. Based on our research, we found that CA inhibits cell apoptosis by promoting the expression of HK-2 and Bcl-2, and inhibiting the expression of Bax. However, we observed no significant difference in XIAP following CA administration.

Autophagy is a conserved eukaryotic cellular degradation that helps maintain cell metabolism. Excessive accumulation of ROS induces autophagy, which eliminates damaged mitochondria and alleviates cellular oxidative stress. Studies have shown that autophagy flow is blocked in the lung tissue of patients with IPF [39]. Stimulating autophagy exerts an antifibrotic effect in the experimental fibrosis model by suppressing oxidative stress [40]. Autophagy is related to plenty of autophagy-related genes, among which LC3 and Beclin1 are important autophagic regulators. PINK1 is critical for mitochondrial clearance by autophagy, and increased PINK1 indicates smooth autophagy flux [41]. p62 is a substrate of autophagy. Thus, a blockage in autophagy may lead to p62 protein accumulation. It was confirmed that kaempferol partially restored the lipidation of LC3 without affecting p62 expression, increased autophagic flux, and attenuated silica-induced pulmonary fibrosis [42]. Ellagic acid could enhance autophagy formation in myofibroblasts mainly by suppressing the Wnt signaling pathway and promoting apoptosis of myofibroblasts [43]. In this study, CA treatment resulted in a significant downregulation of p62, while the expression of Beclin1, PINK1, and transformation of LC3-I to LC3-II were simultaneously activated. TEM is widely regarded as the gold standard for the qualitative detection of autophagy. Studies have demonstrated that increasing numbers of damaged mitochondria were observed in IPF lung tissue [44]. In line with previous research [45], numerous dysmorphic and enlarged mitochondria, and few autophagic vesicles were observed in lung tissues after BLM administration. Treatment with CA was shown to increase the number of autophagic vesicles.

Lysosome is an intracellular organelle that contains a battery of acid hydrolases. Excessive oxidative stress results in destabilization of lysosomal membrane that causes leakage of lysosomal enzymes, which leads to cell apoptosis [46]. Moreover, the fusion of autophagosome and lysosome is the rate-limiting step of autophagy. Lysosomal defects disturb the degradation of autophagic substrates, leading to the accumulation of autophagosomes [47]. Recent studies demonstrated that silica nanoparticles enhanced autophagosome accumulation by impairing lysosomal degradation via acidification inhibition, leading to the apoptosis of AECs, thus resulting in pulmonary fibrosis [48]. However, little attention has been given to lysosomal disorders in pulmonary fibrosis. To date, very few studies have explored the activation of lysosome function in BLM-induced pulmonary fibrosis by naturally products. In this study, we utilized LAMP1 and legumain to measure lysosome function. This study showed that BLM intervention significantly downregulated LAMP1 expression and upregulated legumain expression, which was reversed by CA treatment. These findings suggest that BLM intervention induced lysosomal damage, and that CA treatment may protect lysosomal function and promote autophagic substrate degradation. Considering the lack of extensive lysosomal research in pulmonary fibrosis, additional research on lysosomes should be conducted in future studies.

## 5. Conclusions

In conclusion, this study confirmed that CA improved pulmonary fibrosis induced by BLM in mice, and its mechanism may be related to the inhibition of oxidative stress, activation of the Nrf2/HO-1 pathway, suppression of apoptosis, and upregulation of the autophagy-lysosome pathways. However, in this study, CA was shown to regulate autophagy and apoptosis through multiple pathways [49], and we lack understanding of its potential signaling pathways. Further study would be needed to explore the role of CA in the treatment of idiopathic pulmonary fibrosis.

## Figures and Tables

**Figure 1:** Effects of CA on BLM-induced pulmonary fibrosis. (a, b) Representative images of HE staining (200×) and Masson staining (200×). (c) Immunohistochemistry assays for collagen I (200×). (d–f) Quantitative analysis of inflammation score and Ashcroft score based on HE staining, and collagen area based on Masson staining assays. ^*∗∗*^*P* < 0.01 compared with the NC group; ^#^*P* < 0.05, ^##^*P* < 0.01 compared with the BLM group.

**Figure 2:** Effects of CA on oxidative stress. Total serum levels of (a) MDA, (b) SOD, and (c) TAC as measured through ELISA. (d) Relative mRNA expression of Nrf2. (e) Protein levels of HO-1. (f) Relative density values of HO-1 expression. ^*∗∗*^*P* < 0.01, compared with the NC group, ^#^*P* < 0.05, ^##^*P* < 0.01, compared with the BLM group.

**Figure 3:** Effect of CA on apoptosis-related markers. (a) Bax, (b) Bcl-2, and (c) XIAP mRNA expressions in the lung tissue. (d) Immunohistochemistry assays (200×) for HK-2. ^*∗∗*^*P* < 0.01 compared with the NC group; ^#^*P* < 0.05, ^##^*P* < 0.01, compared with the BLM group.

**Figure 4:** Effects of CA on autophagy. (a) Protein levels of PINK1, Beclin1, p62, and LC3II as measured by western blotting. (b–f) Relative density values showing PINK1, Beclin1, LC3-II, LC3-II/LC3-I, and p62 expression. (g) Representative images of immunohistochemical staining (400×) for p62. ^*∗*^*P* < 0.05, ^*∗∗*^*P* < 0.01, compared with the NC group; ^#^*P* < 0.05, ^##^*P* < 0.01, compared with BLM group.

**Figure 5:** Observation of lung tissue of mice using a transmission electron microscope (20,000×). The white arrowheads indicate autophagosomes, the red arrowheads indicate autolysosomes, and the yellow arrowheads indicate mitochondria.

**Figure 6:** Effects of CA on lysosome injury. (a) Protein levels of LAMP1 and legumain as determined by western blotting. Relative density values showing (b) LAMP1 and (c) legumain expressions. (d) mRNA expression of TFEB. (e) Representative images of immunohistochemical staining (400×) for legumain. ^*∗*^*P* < 0.05, ^*∗∗*^*P* < 0.01, compared with the NC group; ^#^*P* < 0.05, ^##^*P* < 0.01, compared with the BLM group.

## Data Availability

The data are available on request.

## Abbreviations

AECs: Alveolar epithelial cells
BAX: BCL-2-associated X
Bcl-2: B-cell lymphoma-2
BLM: Bleomycin
CA: Calycosin
HE: Hematoxylin-eosin staining
HO-1: Heme oxygenase-1
HK-2: Hexokinase-2
IPF: Idiopathic pulmonary fibrosis
LAMP1: Lysosome-associated membrane protein 1
LC3: Microtubule associated protein 1 light chain 3
MDA: Malondialdehyde
mtROS: Mitochondrial reactive oxygen species
Nrf2: Nuclear factor-erythroid 2-related factor 2
PINK1: PTEN induced putative kinase 1
SQSTM1/p62: Sequestosome
SOD: Superoxide dismutase
TAC: Total antioxidant capacity
TFEB: Transcription factor EB
TEM: Transmission electron microscope
XIAP: X-linked inhibitor of apoptosis protein.
